# Water Quality Prediction Based on SSA-MIC-SMBO-ESN

**DOI:** 10.1155/2022/1264385

**Published:** 2022-08-03

**Authors:** Yan Kang, Jinling Song, Zhuo Lin, Liming Huang, Xiaoang Zhai, Haipeng Feng

**Affiliations:** ^1^School of Mathematics and Information Science & Technology, Hebei Normal University of Science & Technology, Key Laboratory of Ocean Dynamics and Resources and Environments, Hebei Agricultural Data Intelligent Perception and Application Technology Innovation Center, Qinhuangdao 066000, Hebei, China; ^2^School of Business Administration, Hebei Normal University of Science & Technology, Qinhuangdao 066000, China; ^3^CITIC Dicastal Co., Ltd, Qinhuangdao 066000, Hebei, China

## Abstract

Water pollution threatens the safety of human production and life. To quickly respond to water pollution, it is important for water management staff to predict water quality changes in advance. Drawing on the temporality of water quality data, the leaky integrator echo state network (ESN) was introduced to construct the water quality prediction models for dissolved oxygen (DO), permanganate index (CODMn), and total phosphorus (TP), respectively. First, the missing values were filled by the linear trend method of adjacent points, and the outliers were detected and corrected by the *Z*-score method and the linear trend method. Second, the singular spectrum analysis (SSA) was performed to denoise the original monitoring data, such that the predicted data catch up with the real data, and the model accuracy is not affected by the hidden noise in the data. Third, the correlation between water quality indices was measured by the maximum information coefficient (MIC), and the strongly correlated indices were imported to the prediction model. Finally, according to these strong correlation indicators, the water quality prediction models based on multiple features were constructed, respectively, using the offline and online learning algorithms of the ESN. The hyperparameters of the models were optimized through the sequential model-based optimization (SMBO). Experimental results show that the proposed water quality prediction models, namely, SSA-MIC-SMBO-Offline ESN and SSA-MIC-SMBO-Online ESN, predicted DO, CODMn, and TP accurately, providing suitable tools for practical applications.

## 1. Introduction

Water is an important resource for human survival and social development. Unfortunately, water shortage becomes an increasingly severe global problem. One of the major causes of water shortage is water pollution. With limited per-capita water resources, China is deeply troubled by water pollution. According to the 2020 Report on the State of the Ecology and Environment in China (https://www.mee.gov.cn/hjzl/sthjzk/zghjzkgb), 16.6% of the monitored surface water areas in China belong to Classes IV and V in terms of water quality. As the country stepped up the protection of water resources, the focus of water pollution control has shifted from posttreatment to preprevention. To effectively reduce water pollution, it is important to predict the future trend of water quality accurately. The early warning would promote the scientific management of water resources, maintain the sustainability of the ecosystem, and protect human health.

In recent years, many water quality prediction models have been developed based on a dazingly array of technologies, namely, multiple linear regression (MLR) [1], regression tree and support vector regression (SVR) [2], nonlinear least squares (NLS) neural network [3, 4], radial basis function (RBF) neural network [5–7], long short-term memory (LSTM) neural network [8–11], and graph neural network (GNN) [12, 13]. These models greatly advance the prediction of water quality. However, the model performance is affected by various factors in the complex and dynamic system of the water environment, including data quality, input features, prediction algorithm, and selected parameters. Therefore, the existing models should be further improved to forecast water quality more accurately.

This paper constructs the prediction models of water quality indices through comprehensive use of multiple techniques: singular spectrum analysis (SSA), maximum information coefficient (MIC), offline and online learning algorithms of the leaky integrator echo state network (ESN) [14], and sequential model-based optimization (SMBO). First, the original data were smoothed and denoised through the SSA. Next, the correlation between water quality indices was measured by the MIC. Finally, the data on relevant indices were collected from river monitoring stations, and imported to the ESN, the hyperparameters of the network were optimized through the SMBO, and the prediction models were established for dissolved oxygen (DO), permanganate index (CODMn), and total phosphorus (TP), respectively. Experimental results show that the proposed water quality prediction models, namely, SSA-MIC-SMBO-Offline ESN and SSA-MIC-SMBO-Online ESN, forecasted each water quality index accurately and practically.

## 2. Leaky Integrator ESN

The ESN, a novel recurrent neural network (RNN) [14], centers on a large, randomly generated, and sparsely connected reservoir. The only thing that needs to be trained in the network is the output connection weight. Therefore, the ESN boasts the advantages of simple structure and fast training. During the training, the network is not prone to falling to the local optimal trap, a common defect of traditional RNN. In this way, the network weights are always optimized globally.

### 2.1. Network Structure

As shown in Figure 1, the leaky integrator ESN consists of an input layer; a hidden layer, i.e., the reservoir; and an output layer. There are *K* nodes in the input layer, *L* nodes in the output layer, and *N* nodes in the reservoir. At time *t*, the input, the reservoir state, and the output are denoted as *u*(*t*), *x*(*t*), and *y*(*t*), respectively. The *N* × *K* connection weight matrix from the input layer to the reservoir can be expressed as Win. The *N* × *N* connection weight matrix of the reservoir from the current moment to the next moment can be expressed as *W*. The *N* × *L* weight matrix of the feedback connection from the output layer to the reservoir can be expressed as *W*_*fb*_, and the connection is unnecessary. The *L* × (*N* + *K*) connection weight matrix from the reservoir to the output layer can be expressed as *W*_out_. Reservoir, and an output layer. There are *K* nodes in the input layer, *L* nodes in the output layer, and *N* nodes in the reservoir. At time *t*, the input, the reservoir state, and the output are denoted as *u*(*t*), *x*(*t*), and *y*(*t*), respectively. The *N* × *K* connection weight matrix from the input layer to the reservoir can be expressed as Win. The *N* × *N* connection weight matrix of the reservoir from the cu.

The reservoir state *x*(*t*) can be updated based on the current input *u*(*t*) and the reservoir state *x*(*t* − 1) at the previous time, using leaky integrator neurons:

(1) $$\begin{array}{c} x\left(t\right)=\left(1-\alpha \right)x\left(t-1\right)+\alpha f\left(W_{\text{in}}u\left(t\right)+Wx\left(t-1\right)+W_{fb}y\left(t-1\right)\right), \end{array}$$

where *W*_in_, *W*, and *W*_*fb*_ are randomly initialized and fixed before network training; *f* is the activation function; *α* is the leakage rate of the neuron; and *y*(*t* − 1) is the output at the previous time. In this study, the activation function (tanh) and output state equation of the network can be, respectively, expressed as:

(2) $$\begin{array}{c} f\left(x\right)=\frac{e^{x}-e^{-x}}{e^{x}+e^{-x}}, \end{array}$$

(3) $$\begin{array}{c} y\left(t\right)=W_{\text{out}}x\left(t\right). \end{array}$$

### 2.2. Learning Algorithms

In the ESN, the input connection weight matrix *W*_in_ and reservoir connection weight matrix *W* remain unchanged after initialization. Thus, the output connection weight matrix *W*_out_ is the only model parameter that needs to be trained. In essence, the learning process of the ESN is the solving process of *W*_out_. The ESN has two kinds of learning algorithms.

#### 2.2.1. Offline Learning

In the training process of offline learning, to prevent overfitting, *W*_out_ was solved through ridge regression based on the regularization coefficient [15, 16]. This approach adds a regularization term to the objective function. The output weight matrix *W*_out_ can be updated by:

(4) $$\begin{array}{c} W_{\text{out}}={\left(X^{T}X+\lambda I_{N}\right)}^{-1}X^{T}Y, \end{array}$$

where *X* is the state matrix of the reservoir; *λ* is the ridge parameter; *I*_*N*_ is an *N*-dimensional identity matrix; and *Y* is the target output matrix.

#### 2.2.2. Online Learning

Online learning updates the current model with continuously generated new data to make better predictions of future data. The common online learning algorithm is recursive least squares (RLS) [17], which updates *W*_out_ for each time step to minimize the prediction error. By the RLS, the output weight matrix *W*_out_ can be updated by:

(5) $$\begin{array}{c} P\left(t\right)=P\left(t-1\right)-\frac{P\left(t-1\right)x\left(t\right)x^{\text{T}}\left(t\right)P\left(t-1\right)}{1+x^{\text{T}}\left(t\right)P\left(t-1\right)x\left(t\right)}, \end{array}$$

(6) $$\begin{array}{c} W_{\text{out}}\left(t\right)=W_{\text{out}}\left(t-1\right)+\left[d\left(t\right)-y\left(t\right)\right]P\left(t\right)x\left(t\right), \end{array}$$

where *x*(*t*) is the reservoir state; *x*^*T*^(*t*) is the transpose of *x*(*t*); *d*(*t*) is the expected output; *y*(*t*) is the actual output; and *P*(*t*) is the error covariance matrix at time *t*.

In this paper, the ESN using offline learning and that using online learning are denoted as Offline ESN and Online ESN, respectively.

### 2.3. Network Training

According to the principle of the ESN and the input data *u*, the training steps of Offline ESN and Online ESN can be summarized as follows:

#### 2.3.1. Training Steps of Offline ESN

  Step 1: Initialize the reservoir. Configure the relevant parameters; initialize *W*_in_, *W*, *W*_*fb*_, and *W*_out_; and set the reservoir state to the zero vector.
  Step 2: Update and collect the internal state of the reservoir. Drive the reservoir with the input data *u* and update the internal state of the reservoir continuously by formula (1). Note that, to overcome the influence of the initial transient, the state of the previous period is generally abandoned, and the internal state is collected from time *T*.
  Step 3: Calculate W_out_ of the ESN by formula (4).
  Step 4: Calculate the output *y* of the network by formula (3).

#### 2.3.2. Training Steps of Online ESN

  Step 1: initialize the reservoir. Configure the relevant parameters, e.g., reservoir size; initialize *W*_in_, *W*, *W*_*fb*_, and *W*_out_; and set the initial reservoir state to the zero vector.
  Step 2: initialize the relevant parameters in the RLS. Initialize *P*(0) = *ψ* ^−1^*I*, where *ψ* is generally 1 × 10^−8^, and *I* is the identity matrix.
  Step 3: input the sample data *u* into the network, calculate the internal state matrix *x*(*t*) of the ESN by formula (1), update W_out_ by formulas (5) and (6), and solve the corresponding output *y*(*t*) by formula (3).
  Step 4: repeat Step 3 until the input of *u* is completed.

Each connection weight matrix of the ESN can be initialized as follows: each element of the input connection weight matrix *W*_in_ is initialized to random number uniformly distributed in [−0.5, 0.5] and adjusted by the input scaling factor *η*. The reservoir connection weight matrix *W* is initialized to random numbers uniformly distributed in [−0.5, 0.5], discretized according to the sparsity *s*, and readjusted by the target spectral radius *ρ*. The output connection weight matrix *W*_out_ is initialized as a zero matrix.

Considering the principle of the ESN and the need to initialize the connection weight matrices, several parameters need to be set in advance: reservoir size *N*, spectral radius *ρ*, leakage rate *α*, ridge parameter *λ*, input scaling factor *η*, and sparsity *s*. By optimizing the values of these ESN parameters, the accuracy of the prediction model can be significantly improved.

## 3. Data Preprocessing

The original data were collected from the records of the automatic monitoring station of Dongzhen Reservoir in the middle reaches of Mulan river. This reservoir is the drinking water source of over 1.5 million people in Chengxiang District, Licheng District, Xiuyu District, Bei'an Development Zone, and Meizhou Island. Therefore, it is of great significance to precisely predict the water quality at this station.

The water quality at the station is monitored in days. A total of 1,095 pieces of data from 2018 to 2020 were collected, including water temperature (WT), pH, DO, conductivity (Con), turbidity (Tur), ammonia nitrogen (NH_3_–N), CODMn, TP, total nitrogen (TN), and chlorophyll (aChl). The blue-green algae metrics were discarded for the many missing values.

According to the 2020 Report on the State of the Ecology and Environment in China, DO, TP, and CODMn are the main pollution-monitoring indices of surface water in China. Thus, these three water quality indices were selected as prediction objects. Based on the monitoring data of the station, several prediction models were established for the selected indices. The models can apply to other monitoring stations in the Mulan river basin, facilitating the water quality prediction of the entire basin.

The original data contain missing values, outliers, and noise, which may affect the prediction accuracy. To eliminate the effect, some preprocessing operations were implemented on the original data. Specifically, the missing values were filled by the linear trend method of adjacent points, and the outliers were checked and corrected by the *Z*-score method and the linear trend method.

In addition, the SSA [18] was employed to extract signals representing different components of the time series and thus reduced to noise in the time series [19, 20]. The noise reduction solves two common problems: the predicted data fall behind the real data, if the time series data have frequent random fluctuations; the prediction accuracy is suppressed by the implicit noise in the data.

During the SSA, a quarter, i.e., 90 days, was taken as the window length. On this basis, a principal component analysis (PCA) was conducted on the decomposed time series data of water quality. The series of the components, whose cumulative explained variance ratio (EVR) reaches 90%, was taken as the real data, and the remaining components were discarded as noise.

For time series reconstruction, the first 35 components were selected for Con; the first 36 components were selected for NH_3_–N and aChl; the first 37 components were selected for DO, Tur, and pH; the first 38 components were selected for TP and CODMn; and the first 39 components were selected for WT and TN. Figures 2–4 display the time series of DO, CODMn, and TP before and after reconstruction. Compared with the original time series, the reconstructed time series contain no extreme values and have obvious cycle and trend. Therefore, the reconstructed data were adopted as the real data for water quality indices.

The denoised water quality data were further normalized through max-min normalization, which maps sample values to the interval [0, 1]:

(7) $$\begin{array}{c} X^{\prime }=\frac{X-X_{\min}}{X_{\max}-X_{\min}}, \end{array}$$

where *X*_min_ and *X*_max_ are the minimum and maximum values in the sample, respectively; *X* is the original value of the sample.

## 4. MIC-Based Correlation Analysis of Water Quality Indices

The water environment is a complex dynamic system affected by many factors. The system faces both material changes and energy exchanges. Besides, there may be some correlations between water quality indices. The indices related to the prediction index could be used together as input features. Drawing on the mutual information theory, this section analyzes the correlation between water quality indices.

The mutual information of a random variable pair (*X*, *Y*) was adopted to describe the amount of information about variable *Y* contained in variable *X*:

(8) $$\begin{array}{c} I\left(X;Y\right)=\sum_{x\in X}\sum_{y\in Y}p\left(x,y\right)\log\frac{p\left(x,y\right)}{p\left(x\right)p\left(y\right)}, \end{array}$$

where *p*(*x*, *y*) is the joint distribution of *X* and *Y*; *p*(*x*) and *p*(*y*) are the marginal distributions of *X* and *Y*, respectively.

The MIC [21] measures the correlation between variables. The coefficient falls between 0 and 1. The greater the value, the stronger the correlation [22]. MIC can be calculated by:

(9) $$\begin{array}{c} \text{MIC}\left(x,y\right)=\underset{ij<B}{\max}\frac{I\left[D\left(x,y\right)\right]}{\log\;\min\left(x,y\right)}, \end{array}$$

where *ij* < *B* is the constraint of the total number of grids; *B* is set to the power of *θ* of the size of dataset *D*. Relevant studies show that the optimal *θ* is 0.6, when the dataset size is between 1,000 and 2,500 [23].

Unlike mutual information, MIC can solve continuous variables at a high accuracy. With sufficient samples, MIC can detect a wide range of linear and nonlinear relationships between variables, making it possible to mirror the degree of correlation between water quality indices [24]. The specific value of MIC can be determined as follows:

  Step 1: For the two given random variables (*X*, *Y*), rearrange the data elements of each variable in a certain order, producing an ordered pair set D(*X*, *Y*).
  Step 2: Mesh the scatterplot of the ordered pair set *D*(*X*, *Y*) into *i* columns and *j* rows (the values of *i* and *j* are given) and then calculate *I*(*X*; *Y*).
  Step 3: Normalize the obtained mutual information.
  Step 4: Select different combinations of *i* and *j* to divide the random variables, and then find out the maximum mutual information (i.e., MIC) for each division method.

Here, the MIC analysis algorithm is adopted to analyze the correlation between DO, CODMn, and TP of Dongzhen Reservoir; the three target indices; and three other water quality indices (Table 1). The results in Table 2 show that the three other indices are strongly correlated with the three target indices. Thus, these three indices were taken as the common input features of the target indices.

## 5. SSA-MIC-SMBO-ESN Water Quality Prediction Model

The transmission and diffusion of pollutants in the upstream affect the concentration of pollutants in the downstream. Considering this effect, the data on water quality indices were collected from four inflow river-monitoring stations (Changtaixi Tukeng Reservoir, Dongtaixi Dongtai Village, Dulixi Xiashan Village, and Juxi Guoxi Village) and added to the ESN as input features. For each target index, a total of eight features were imported to the ESN.

To ensure the timeliness of the forecast, a 3-day forecast model was constructed for each index. The input features are denoted as *t* − *w* + 1 to *t*, and the outputs (predicted values) are denoted as *t* + 1, *t* + 2, and *t* + 3. Then, the ESN has *K* = 8*w* input nodes and *L* = 3 output nodes. Note that *w* is a dynamic optimization parameter.

To fully mine the information of each time series, the monitoring data of the first 1,045 days were organized into the training set, and those of the last 50 days into the test set. In addition, the first 45 states were discarded to eliminate the influence of the initial state.

### 5.1. SMBO-Based Hyperparameter Optimization

According to the network training process, the following hyperparameters of the ESN need to be optimized, namely, reservoir size *N*, spectral radius *ρ*, leakage rate *α*, ridge parameter *λ*, input scaling factor *η*, sparsity *s*, and window length *w*. These hyperparameters were optimized to build our water quality prediction model. The optimization of hyperparameters essentially aims to improve the loss function in the configuration space. Suppose the optimization problem pursues minimization, then, hyperparameter optimization can be expressed as:

(10) $$\begin{array}{c} x^{*}=\text{arg}\underset{x\in X}{\text{min}}f\left(x\right), \end{array}$$

where *f*(*x*) is the objective function to be minimized; *x* is the set of hyperparameters (*N*, *ρ*, *α*, *λ*, *η*, *s*, and *w*); *X* is the hyperparameter domain; and *x*^*∗*^ is the set of the smallest hyperparameters. *x* can take any value in the domain *X*.

The evaluation of the objective function is generally costly, and the manual or grid search parameter tuning method is time-consuming. By contrast, Bayesian optimization greatly improves the search efficiency, as it approximates the objective function with a low-cost adaptive surrogate model. Bayesian optimization aims to model the objective function, according to the existing *N* groups of experimental results *H* = {*x*_*n*_, *y*_*n*_} (*n* ∈ [1, *N*], where *y*_*n*_ is the observed value of *f*(*x*_*n*_)), and to calculate *p*(*y*|*x*, *H*) (i.e., the surrogate model) of *y*. The surrogate model uses the tree-structured Parzen estimator (TPE). The value of *p*(*y*|*x*) can be calculated by:

(11) $$\begin{array}{c} p\left(y|x\right)=\frac{p\left(x|y\right)p\left(y\right)}{p\left(x\right)}. \end{array}$$

Sufficient sampling is critical to make the surrogate model approach the objective function. To reduce the cost of sample generation, it is favorable to control the sample size being used. Hence, formula (9) was adopted to evaluate the profit brought by a sample to the surrogate model. The larger the profit, the closer the updated surrogate model will be to the objective function. Generally, the profit can be measured by expected improvement (EI):

(12) $$\begin{array}{c} \text{EI}\left(x,H\right)=\int_{-\infty }^{\infty }\max\left(y*-y,0\right)p\left(y|x,H\right)\text{d}y, \end{array}$$

where *y*^*∗*^ = min{*y*_*n*_, 1 ≤ *n* ≤ *N*} is the optimal value in the current existing samples. The EI refers to the expectation that the value *y* of a sample *x* under the current surrogate model *p*(*y* | *x*, *H*) exceeds the best result *y*^*∗*^.

The SMBO is a specific algorithm to implement Bayesian optimization [25]. The algorithm 1can be described as follows:

For hyperparameter optimization by the SMBO, the search space and step size of each parameter were configured as shown in Table 3, and the number of iterations LT was set to 5,000.

### 5.2. Performance Metrics

The predictive power of our water quality prediction models was evaluated by root mean square error (RMSE), mean absolute percentage error (MAPE), and Nash–Sutcliffe efficiency (NSE) [26, 27]. Among them, the NSE specifically verifies the simulation results of the hydrological model. The value of NSE falls between 0 and 1. The larger the value, the stronger the prediction ability of the model. The RMSE, MAPE, and NSE can be, respectively, calculated by:

(13) $$\begin{array}{c} \text{RMSE}=\sqrt{\frac{1}{n}\sum_{i=1}^{n}{\left(y_{i}-{\hat{y}}_{i}\right)}^{2}}, \end{array}$$

(14) $$\begin{array}{c} \text{MAPE}=\frac{100\%}{n}\sum_{i=1}^{n}\left|\frac{{\hat{y}}_{i}-y_{i}}{y_{i}}\right|, \end{array}$$

(15) $$\begin{array}{c} \text{NSE}=1-\frac{\sum_{i=1}^{n}{\left(y_{i}-{\hat{y}}_{i}\right)}^{2}}{\sum_{i=1}^{n}{\left(y_{i}-\bar{y}\right)}^{2}}, \end{array}$$

where *y*_*i*_ is the target output; *ŷ*_*i*_ is the network output; and *ȳ* is the mean of the target output.

### 5.3. Construction of the SSA-MIC-SMBO-Offline ESN Model

Offline learning, also known as batch learning, inputs all sample data at once to train the model. During training, the data on the eight input features for each target index were imported to the Offline ESN. The hyperparameters of the Offline ESN were optimized by SMBO.  Table 4 displays the optimization results. On this basis, the authors established the SSA-MIC-SMBO-Offline ESN prediction model for each water quality index.  Table 5 shows the index values obtained by verifying each prediction model on the test set. Figures 5–7 compare the predicted value with the actual value of each prediction model.

As shown in Table 5 and Figures 5–7, the SSA-MIC-SMBO-Offline ESN prediction models of DO, CODMn, and TP generally performed well. In particular, the predicted value and actual value basically overlapped in the first 2 days. Thus, the SSA-MIC-SMBO-Offline ESN 3-day prediction model constructed for each water quality index can meet the requirements of practical application. However, the predicted values of the three indices on the second and third days gradually deviated from the actual values, with the deterioration of each evaluation index. This means the prediction effect weakens over the time. Specifically, the prediction indices of all prediction models were good on the first day, where the NSE values were all above 0.98, indicating that the prediction models have a high prediction accuracy for the next day. The NSE values of the prediction indices were all around 0.9 on the second day (only the NSE of the CODMn was slightly low), suggesting that the accuracy on the second day also maintains a high level. The NSE values of the prediction indices of each prediction model reached about 0.8 on the third day, and the values of other evaluation indices were also within the acceptable range. Hence, the prediction effect on the third day can also meet the application requirements.

### 5.4. Construction of the SSA-MIC-SMBO-Online ESN Model

The data on the eight input features for each target index were imported to the Online ESN. The hyperparameters of the Online ESN were optimized by SMBO.  Table 6 displays the optimization results. On this basis, the authors established the SSA-MIC-SMBO-Online ESN prediction model for each water quality index.  Table 7 shows the index values obtained by verifying each prediction model on the test set. Figures 8–10 compare the predicted value with the actual value of each prediction model.

Experimental results show that the SSA-MIC-SMBO-Online ESN prediction models of DO, CODMn and TP output ideal prediction index values and prediction curves in the first two days. On the first day, the prediction index values of each prediction model were very good. The RMSEs were around 0.01, the MAPEs were within 0.09, and the NSEs were above 0.985, indicating that the prediction models have a very high prediction accuracy for the next day. On the second day, the RMSEs of the prediction indices were all around 0.04, and the NSE values were around 0.9 (only the NSE value of the CODMn was slightly low), indicating that the accuracy can also reach a high level on the second day. On the third day, the RMSEs of the prediction models reached about 0.06, the NSEs stood at about 0.8, and the MAPEs were within the acceptable range. Overall, the prediction effect on the third day is significantly lower than that on the previous two days, but it can still meet the application requirements. It can also be seen that, on the first day, the prediction curves of the three water quality indices largely overlapped the actual curves. On the second and third days, the prediction curves gradually deviated from the real curves, and exhibited some oscillations. However, the two sets of curves obeyed consistent trends. In general, the SSA-MIC-SMBO-Online ESN 3-day prediction models for DO, CODMn and TP achieved desirable performances, indicating that the model is feasible to predict each water quality index.

### 5.5. Discussion

From the experimental results, it is easy to find that the SSA-MIC-SMBO-Offline ESN and SSA-MIC-SMBO-Online ESN water quality prediction models can basically forecast the values of DO, CODMn, and TP. Further comparison shows that the SSA-MIC-SMBO-Online ESN model had better evaluation indices than the SSA-MIC-SMBO-Offline ESN model. On the first day, the three water quality indices predicted by SSA-MIC-SMBO-Online ESN were about 0.001 smaller than those predicted by SSA-MIC-SMBO-Offline ESN, while the NSEs were 0.002 larger. On the second day, the RMSE of DO predicted by SSA-MIC-SMBO-Online ESN was 0.0015 smaller than that of DO predicted by SSA-MIC-SMBO-Offline ESN, while the NSEs were 0.013 larger. The other two indices predicted by SSA-MIC-SMBO-Online ESN were also better than those predicted by SSA-MIC-SMBO-Offline ESN in the same period. Overall, the SSA-MIC-SMBO-Online ESN prediction models were more accurate than the SSA-MIC-SMBO-Offline ESN prediction models and more suitable for projecting the dynamics changes in water quality data.

Concerning the commonality of the prediction effects of the SSA-MIC-SMBO-Offline ESN or SSA-MIC-SMBO-Online ESN on the three target indices, the TP prediction model had the best index value than DO and CODMn prediction models in the same period. The DO prediction model outperformed the CODMn prediction model in terms of index value and prediction effect. Meanwhile, the CODMn prediction model had the lowest accuracy. Judging by the performance of the offline and online prediction models of the three indices, it can be observed that the prediction performance is closely related to the data features of the target indices. The prediction performance is good when the index data are clear and not frequently changeable. But the prediction accuracy tends to be low when the index data (e.g., CODMn) fluctuate greatly and frequently, making it difficult for any prediction model to capture the laws and features of the data. This is also the limitation of this prediction method. Therefore, the performance of the prediction models can be further enhanced by inputting more relevant features and expanding the training set.

## 6. Conclusions

Based on the important water quality indices related to water pollution, this paper separately establishes ESN-based offline and online water quality prediction models by using singular spectrum analysis algorithm, maximum mutual information coefficient, echo state network, and sequential model optimization algorithm. These models achieve good prediction results, and it can be seen from the above experimental results that the SSA-MIC-SMBO-Online ESN prediction models are more accurate than the SSA-MIC-SMBO-Offline ESN prediction models and more suitable for projecting the dynamics changes in water quality data.

The water environment is a complex system affected by many factors. The change of each water quality index is related to various factors rather than the water environment alone. For instance, the DO in the water body depends on climate factors such as water temperature, air pressure, and light. Therefore, the prediction of water quality indices must consider multiple influencing factors, as well as the correlation between water quality indices and meteorological factors/pollution sources. In the future, our research team will improve the proposed prediction models by supplementing various relevant data and further optimize the ESN algorithm from multiple perspectives: improving the reservoir generation approach, improving the initialization of connection weights of the reservoir, optimizing these weights, streamlining the reservoir topology, rationalizing neuron selection, and so on. In addition, LSTM and its improved algorithms will be considered for water quality prediction work in this study.

## Figures and Tables

**Figure 1:** Structure of the leaky integrator ESN.

**Figure 2:** Reconstructed series of DO.

**Figure 3:** Reconstructed series of CODMn.

**Figure 4:** Reconstructed series of TP.

**Figure 5:** Effect of SSA-MIC-SMBO-Offline ESN 3-day prediction model for DO.

**Figure 6:** Effect of SSA-MIC-SMBO-Offline ESN 3-day prediction model for CODMn.

**Figure 7:** Effect of SSA-MIC-SMBO-Offline ESN 3-day prediction model for TP.

**Figure 8:** Effect of SSA-MIC-SMBO-Online ESN 3-day prediction model for DO.

**Figure 9:** Effect of SSA-MIC-SMBO-Online ESN 3-day prediction model for CODMn.

**Figure 10:** Effect of SSA-MIC-SMBO-Online ESN 3-day prediction model for TP.

**Algorithm 1:** SMBO algorithm.

**Table 1:** Input features of prediction model.

Predictive evaluation indicators	Input features
DO	DO, pH, NH_3_–N, Con
CODMn	CODMn, WT, Tur, aChl
TP	TP, Tur, pH, Con

**Table 2:** Results of MIC correlation analysis.

	WT	pH	DO	Tur	NH_3_–N	CODMn	TP	TN	aChl	Con
DO	0.210	0.497	1	0.219	0.310	0.131	0.192	0.148	0.245	0.283
CODMn	0.363	0.199	0.131	0.361	0.143	1	0.171	0.249	0.316	0.314
TP	0.168	0.223	0.192	0.217	0.192	0.171	1	0.158	0.156	0.232

**Table 3:** Parameter space optimized by SMBO.

Parameter	Range	Step size
*N*	[50, 400]	10
Ρ	[0.1, 1.5]	0.1
Α	[0.01, 0.1]	0.01
Η	[0.1, 1]	0.1
*s*	[0.01, 0.1]	0.01
*λ*	[1*e* − 5, 1]	Increase 10 times each time
*w*	[3, 15]	1

**Table 4:** Hyperparameter optimization results of the SSA-MIC-Offline ESN 3-day prediction model.

Evaluation index	Model parameters
DO	*N* = 140, *ρ* = 0.63, *α* = 0.23, *λ* = 1.*E* − 04, *η* = 0.1, *s* = 0.06, *w* = 5
CODMn	*N* = 170, *ρ* = 0.61, *α* = 0.49, *λ* = 1.*E* − 04, *η* = 0.8, *s* = 0.01, *w* = 10
TP	*N* = 70, *ρ* = 1.29, *α* = 0.63, *λ* = 1.*E* − 02, *η* = 0.4, *s* = 0.06, *w* = 5

**Table 5:** Index values of SSA-MIC-SMBO-Offline ESN 3-day prediction model.

Water quality indicator	Prediction step	RMSE	MAPE	NSE
DO	1	0.0091	0.059	0.992
	2	0.0314	0.175	0.906
	3	0.0608	0.603	0.824

CODMn	1	0.0194	0.092	0.984
	2	0.0607	0.356	0.887
	3	0.0946	0.649	0.753

TP	1	0.0124	0.028	0.991
	2	0.0341	0.080	0.938
	3	0.0556	0.135	0.840

**Table 6:** Hyperparameter optimization results of the SSA-MIC-Online ESN 3-day prediction model.

Evaluation index	Model parameters
DO	*N* = 50, *ρ* = 0.05, *α* = 0.91, *η* = 0.7, *s* = 0.05, *w* = 7
CODMn	*N* = 130, *ρ* = 0.77, *α* = 0.31, *η* = 0.9, *s* = 0.04, *w* = 14
TP	*N* = 50, *ρ* = 1.32, *α* = 0.98, *η* = 0.2, *s* = 0.05, *w* = 4

**Table 7:** Index values of the SSA-MIC-SMBO-Online ESN 3-day prediction model.

Water quality indicator	Prediction step	RMSE	MAPE	NSE
DO	1	0.0087	0.058	0.993
	2	0.0299	0.153	0.919
	3	0.0503	0.484	0.846

CODMn	1	0.0187	0.089	0.986
	2	0.0573	0.332	0.897
	3	0.0814	0.506	0.786

TP	1	0.0102	0.022	0.994
	2	0.0328	0.076	0.941
	3	0.0527	0.118	0.867

## Data Availability

The data used to support the findings of this study are available from the corresponding author upon request.
